RETRACTED

# The Tumor-Suppressive MicroRNA-135b Targets c-Myc in Osteoscarcoma

**DOI:** 10.1371/journal.pone.0102621

**Published:** 2014-07-15

**Authors:** Zheng Liu, Guangwu Zhang, Jian Li, Jiabang Liu, Pengfeng Lv

**Affiliations:** Department of Orthopedic Surgery, Peking University Shougang Hospital, Beijing, China; H.Lee Moffitt Cancer Center & Research Institute, United States of America

## Abstract

Osteosarcoma is the most common primary tumor of the bone. It leads to many deaths because of its rapid proliferation and metastasis. Recent studies have shown that microRNAs are important gene regulators that are involved in various cancer-related processes. In this study, we found that miR-135b was down-regulated in both osteoscarcoma patient tumor tissues and osteoscarcoma cell lines in comparison to paired adjacent non-tumor bone tissue. We observed that a lower level of miR-135b was associated with metastasis. The ectopic expression of miR-135b markedly suppressed osteoscarcoma cell proliferation, migration, and invasion. Conversely, the inhibition of miR-135b expression dramatically accelerated cell proliferation, migration, and invasion. The forced expression of miR-135b in osteosarcoma cells resulted in a significant reduction in the protein level of c-Myc and repressed the activity of a luciferase reporter that contained the 3′-untranslated region of the c-Myc mRNA. These effects were abolished by the mutation of the predicted miR-135b-binding site, which indicates that c-Myc may be a miR-135b target gene. Moreover, the ectopic expression of c-Myc partially reversed the inhibition of cell proliferation and invasion that was caused by miR-135b. These data therefore suggest that miR-135b may function as a tumor suppressor to regulate osteosarcoma cell proliferation and invasion through a mechanism that targets the c-Myc oncogene. These findings indicate that miR-135b may play a role in the pathogenesis of osteosarcoma.

## Introduction

Osteosarcoma is the most common primary malignancy, and it arises primarily in the metaphysis of the long bones in adolescents and young adults [1], [2]. It is primarily present around regions with active bone growth and repair, such as the knee joint, lower femur, and upper tibia [3]. Osteosarcoma is locally destructive and has a high metastatic potential [4]. Despite the rapid development of treatment strategies, curing patients with osteosarcoma is still difficult [5]. Patients who are treated with amputation alone often die of pulmonary metastasis within one year [6]. It is therefore necessary to investigate the fundamental molecular mechanisms that underlie the histological heterogeneity, drug resistance, and development of metastasis to identify novel markers for the diagnosis, prognosis, and treatment of patients with this disease.

RETRACTED

MicroRNAs (miRNAs) are a family of small, non-coding, endogenous RNA molecules that post-transcriptionally regulate target gene expression by sequence-specific base pairing with mRNAs [7]. Growing evidence has suggested that miRNAs play important roles in many biological processes, including differentiation, proliferation, apoptosis, cell cycle, migration and invasion [8]. Previous results have suggested that miRNAs are involved in human carcinogenesis. Furthermore, the aberrant expression of specific miRNAs has been found to be associated with the development and clinical outcomes of various cancers [9]–[11]. However, deregulated miRNAs and their roles in tumorigenesis are still largely unknown.

It has also been reported that miR-135b is involved in the progression of several types of cancer [12]. For example, miR-135b has been found to be overexpressed in colon, breast, and lung cancer [12]–[16]. However, the expression and function of miR-135b is still unknown in osteosarcoma. In the present study, we found that miR-135b was down-regulated in osteosarcoma cell lines and primary tumor samples. miR-135b was further identified to be a tumor suppressor because the restoration of miR-135b expression in osteosarcoma cell lines reduced cell proliferation and suppressed cell migration and invasion. The important anti-invasion molecule c-Myc was identified to be a novel and direct target of miR-135b. Our data suggest that the pro-invasion function of miR-135b occurs primarily through targeting c-Myc expression. Thus, our data suggest important roles for miR-135b in osteosarcoma pathogenesis and indicate its potential application in cancer therapy.

## Materials and Methods

### Ethics Statement

All of the patients (or patients’ parents on behalf of the children) agreed to participate in the study and gave written informed consent. Both this study and consent were approved by the Ethics Committee of Peking University Shougang Hospital and complied with the Declaration of Helsinki.

### Patient and tumor samples

Osteosarcomas and morphologically normal tissues (located >3 cm away from the tumor) were obtained between 2008 and 2012 from 80 osteosarcoma patients who were undergoing surgery at the Department of Orthopedic Surgery at The First Affiliated Hospital of Harbin Medical University. Tissue samples were cut into two parts, and one section was fixed with 10% formalin for histopathological diagnosis. The other section was immediately snap-frozen in liquid nitrogen and then stored in liquid nitrogen until it was needed for RNA extraction. None of the patients received radiotherapy or chemotherapy before surgery. The use of the tissue samples for all of the experiments was approved by each of the patients and by the Ethics Committee of Peking University Shougang Hospital. The characteristics of the patients are described in Table S1.

RETRACTED

### Cell lines and cell culture

The following human cell lines were used in this study: MG-63 (14 year’s old, male), U2OS (15 year’s old, female), SOSP-9607 (17 year’s old, male), and SAOS-2 (11 year’s old, female). These cell lines were purchased from the Cell Resource Center of the Institute of Basic Medical Sciences at the Chinese Academy of Medical Sciences and the Peking Union Medical College (Beijing, China) and were propagated in Dulbecco’s modified Eagle’s medium (Gibco; Invitrogen; Life Technologies, Germany) that was supplemented with 10% fetal bovine serum (GIBCO, NY, USA), streptomycin (100 µg/ml), and penicillin (100 U/ml).

### Cell transfection

The miR-135b mimics, inhibitor and scrambled (which was non-homologous to the human genome) miRNA were synthesized by GenePharma (Shanghai, China) and were transfected into the cells with a final oligonucleotide concentration of 20 nmol/L. All of the cell transfections were performed with DharmaFECT1 reagent (Dharmacon, TX, USA), according to the manufacturer’s instructions. For each cell transfection, two or three replicate experiments were performed.

### TaqMan RT-PCRs for miRNA expression

Total RNA was extracted from the cells and tissues with Trizol reagent (Invitrogen, Calsbad, CA, USA). MicroRNAs were quantitated by real-time PCR using TaqMan MicroRNA Assays (Invitrogen, USA). First-strand complementary DNA (cDNA) synthesis was carried out with 1 µg of total RNA in a 12-µl final volume that contained 2 M of the stem-loop primer and 10 mM dNTP Mix (Invitrogen, USA). The mix was incubated at 65°C for 5 min and then mixed with 5x RT buffer, 0.1 M DTT, 200 U/µl of MultiScribe reverse transcriptase, and 40 U/µl of RNase inhibitor (Invitrogen, USA). The mix was incubated at 37°C for 55 min, at 70°C for 15 min, and then held at −20°C. Real-time PCR was performed by following a standard TaqMan PCR protocol. The 20-µl PCRs included 1 µl of RT product, 1x Universal TaqMan Master Mix and 1x TaqMan probe/primer mix (Invitrogen, USA, Table S2). All RT reactions, including reactions containing no-template controls, were run in triplicate. All mRNA quantification data were normalized to U6 expression. The relative amount of transcript was calculated using the comparative C_t_ method. All miRNA quantification data were normalized to U6. All mRNA quantification data were normalized to GAPDH.

### Cell proliferation assays

Cells were incubated in 10% CCK-8 (Dojindo; Kumamoto, Japan) that was diluted in normal culture medium at 37°C until the visual color conversion occurred. Proliferation rates were determined at 0, 24, 48, 72, and 96 hours after transfection.

RETRACTED

### Cell migration and invasion assays

Wound-healing assays were performed to assess cell migration. An artificial wound was created 24 hours after transfection by using a 200-µL pipette tip on the confluent cell monolayer. Mitomycin C was then added to the culture wells. To visualize cell migration and wound healing, images were taken at 0, 24, and 48 hours.

Invasion assays were performed by examining the ability of cells to pass through a Matrigel-coated membrane matrix (BD Biosciences). Cells were seeded 24 hours after transfection onto a Matrigel-coated membrane matrix that was present in the insert of a 24-well culture plate. Fetal bovine serum was added to the non-invading cells that were removed. Invasive cells that were located on the lower surface of the chamber were stained with 0.1% crystal violet (Sigma) and were then counted.

### Dual luciferase assays

Cells were co-transfected with 0.4 µg of the reporter construct, 0.2 µg of the pGL-3 control vector, and either miR-135b or a negative control. Cells were harvested 24 h post-transfection and then assayed with the Dual Luciferase Assay (Promega, WI, USA), according to manufacturer’s instructions. Firefly luciferase values were normalized to the Renilla signal, and the ratio of the Firefly/Renilla values were reported. All of the transfection assays were carried out in triplicate.

### Western blot analysis

Western blot analysis was carried out using standard methods. Proteins were separated by 10% SDS-PAGE and then transferred to PVDF membranes (Amersham, Buckinghamshire, UK). Membranes were blocked overnight with 5% non-fat dried milk and incubated for 2 h with anti-c-Myc antibody (Abcam, England) at a 1∶1000 dilution or with anti-GAPDH antibody (Proteintech, Chicago, USA) at a 1∶50000 dilution. After washing with TBST (10 mM Tris pH 8.0, 150 mM NaCl, and 0.1% Tween-20), the membranes were incubated for 2 h with a goat anti-rabbit antibody (zsgb-bio, Beijing, China) at either a 1∶5000 dilution or a 1∶50000 dilution.

### Rescue assays of c-Myc gene expression

The full-length c-Myc cDNA (which included the ORF and 3′UTR) was PCR-amplified and cloned into the pcDNA3.1 vector to generate the pcDNA-c-Myc constructs that were used in the rescue assays. MG-63 cells in 6-well plates were first transfected with either the miR-135b or a scrambled dsRNA (20 nM). After 24 h in culture, these cells were then co-transfected with miR-135b (20 nM) and 2 µg of the pcDNA-c-Myc plasmid DNA or with miR-135b (20 nM) and 2 µg of the pcDNA empty vector plasmid. Cells were harvested at the indicated time points after hemin addition and were assayed as required.

RETRACTED

### Statistical analysis

Each experiment was repeated at least three times. Statistical analyses were performed using SPSS 15.0. Data are presented as the mean ± standard deviation. Statistical analyses were performed with either an analysis of variance (ANOVA) or Student’s t-test, and the statistical significance level was set at α = 0.05 (two-side).

## Results

### miR-135b Is down-regulated in osteosarcoma cell lines and tissues

The expression of miR-135b was examined in four human osteosarcoma cells lines (MG-63, U2OS, SOSP-9607, and SAOS-2) and in four osteosarcoma tissues and adjacent non-neoplastic tissues (Fig. 1A). The osteosarcoma cells lines exhibited a significantly lower expression of miR-135b compared to the four pairs of adjacent tissues. Furthermore, the expression of miR-135b in the osteosarcoma tissues was clearly decreased in comparison to the adjacent tissues (Fig. 1A).

**Figure 1:** The expression of miR-135b in human osteosarcoma cell lines and tissues. (A) The expression of miR-135b in four human osteosarcoma cell lines (MG-63, U2OS, SOSP-9607, and SAOS-2), four primary tissues (C) and adjacent non-neoplastic tissues (N) were analyzed by using real-time PCR. (B) miR-135b was detected in 80 osteosarcoma patients by real-time PCR. Data are presented as the log_2_ fold-change in GC tissues relative to the adjacent non-tumor tissues. (C) The expression of miR-135b in the osteosarcoma tissues was lower than in the adjacent non-tumor tissues (p<0.01). (D) The expression of miR-135b in the metastatic osteosarcoma tissues was lower than in the non-metastases tissues. Experiments were performed three times. U6 snRNA was used as the endogenous control. All data were analyzed using a t-test and are shown as the mean±SD (*p<0.05, **p<0.01 and ***p<0.001).

### The expression of miR-135b in clinical osteosarcoma patients and a correlation analysis with clinicopathological characteristics

Among the 80 osteosarcoma samples, miR-135b was down-regulated in 71 cases (71/80, 88.8%) in comparison to the adjacent tissues (Fig. 1B). However, miR-135b was up-regulated in 9 cases (9/80, 11.2%). In general, the expression of miR-135b in osteosarcoma tissues was significantly lower than in the adjacent tissues (Fig. 1C, p<0.001). The expression of miR-135b in the metastatic osteosarcoma tissues was significantly lower than in the non-metastatic tissues (p<0.001, independent-samples t-test).

### miR-135b inhibits osteosarcoma cell proliferation

To study the role of miR-135b in the development of osteosarcoma, MG-63 cells were transfected with both a miR-135b mimic and inhibitor. Both miRNAs showed a high level of transfection efficiency (Fig. 2A). CCK-8 proliferation assays showed that the cell growth rate was reduced in the miR-135b mimic-transfected MG-63 cells compared with either the scrambled miRNA-transfected cells or the untreated cells (Fig. 2B). In contrast, the miR-135b inhibitor significantly accelerated the cell proliferation of the MG-63 cells. The proliferative effects of miR-135b were further confirmed by examining ki-67 expression. As shown in Fig. 2C and D, there were significant decreases in the protein and mRNA levels of ki-67 in the cells that were transfected with the miR-135b mimic in comparison to the control and untreated groups. However, the miR-135b inhibitor significantly increased the expression of ki-67 at both the protein and mRNA levels.

RETRACTED

**Figure 2:** miR-135b inhibits osteosarcoma cell proliferation. (A) Examination of mir-135b expression in MG-63 cells that were transfected with 20 nmol/L of the indicated miRNA. Samples were analyzed 48 h after transfection. (B) Growth assays were performed 0 h, 24 h, 48 h, 72 h, and 96 h after transfection. (C) The expression of ki-67 mRNA was detected by real-time RT-PCR. The MG-63 cells were transfected with 20 nmol/L of the indicated miRNA and were analyzed 48 h later. GAPDH was used as the endogenous control. (D) The expression of ki-67 protein was detected by Western blotting. The MG-63 cells were transfected with 20 nmol/L of the indicated miRNA and were analyzed 48 h later. GAPDH was used as the loading control. Experiments were performed three times. The bars represent the mean±SD (*p<0.05, **p<0.01 and ***p<0.001).

### miR-135b inhibits cell migration and invasion in vitro

To analyze the role of miR-135b in cell migration and invasion, which are key determinants of malignant progression and metastasis, wound healing and trans-well assays were performed with MG-63 cells. The cells that were treated with the miR-135b mimic were distinctively less migratory than the scrambled control or untreated cells at the 12, 24, and 36 hour time points following scratching (Fig. 3A). In contrast, the miR-135b inhibitor significantly accelerated the cell migration of the MG-63 cells. Furthermore, we conducted cell invasion Matrigel assays and then stained the invaded cells to measure the directional invasion ability of the cells after ectopically expressing miR-135b in MG-63 cells. The invasiveness of the cells that were transfected with the miR-135b mimic was dramatically decreased compared with the scrambled control and untreated cells. However, the miR-135b inhibitor significantly increased the invasion of the MG-63 cells (Fig. 3B).

RETRACTED

**Figure 3:** The influence of miR-135b on osteosarcoma cell migration and invasion. (A) Wound healing assays were carried out with MG-63 cells after treatment with the indicated miRNA. The relative ratios of wound closures per field is shown. (B) Trans-well analysis of MG-63 cells after treatment with the indicated miRNA. The relative ratios of invasive cells per field is shown. The bars represent the mean±SD (*p<0.05, **p<0.01 and ***p<0.001).

### miR-135b targets c-myc in osteosarcoma cells

As predicted by PicTar, there was complementarity between has-miR-135b and the c-Myc 3′UTR (Fig. 4A). miR-135b overexpression reduced the protein but not the mRNA levels of c-Myc in osteosarcoma cells (Fig. 4B and D). The effects of miR-135b on the translation of c-Myc mRNA into protein was then assessed by using a luciferase reporter assay (Fig. 4C). miR-135b overexpression remarkably reduced the luciferase activity of the reporter gene with the wild-type construct but not with the mutant c-Myc 3′UTR construct, which indicates that miR-135b directly targeted the c-Myc 3′UTR.

**Figure 4:** c-Myc is a direct target of miR-135b. (A) A schematic representation of the c-Myc 3′UTR that shows the putative miRNA target site. (B) Real-time PCR analysis shows that miR-135b does not alter the mRNA level of c-Myc. (C) Luciferase activities of the wild-type (WT-UTR) and mutant (MUT-UTR) constructs. (D) c-Myc protein expression in osteosarcoma cells that were transfected with 50 nmol/L of the indicated miRNA. Values are presented as the mean±SD.

### Overexpression of c-Myc impairs the miR-135b-induced inhibition of proliferation and invasion in MG-63 cells

To assess the regulation of miR-135b on c-Myc expression, the protein level of c-Myc was analyzed in eight miR-135b-down-regulated osteosarcoma tissues. c-Myc was up-regulated in seven of the osteosarcoma tissues (Fig. 5C). We then performed rescue experiments to further validate that the targeting of c-Myc was involved in the anti-tumor properties of miR-135b in osteosarcoma cells. The c-Myc expression vector pcDNA3.1-c-Myc was used to restore c-Myc expression. The inhibition of cell proliferation and invasion upon overexpression of miR-135b was significantly attenuated by the re-introduction of c-Myc (Fig. 5A and B).

**Figure 5:** c-Myc is required for miR-135b-directed osteosarcoma cell proliferation and invasion. (A) Western blot analysis of c-Myc in MG-63 cells that were co-transfected with either a miR-135b mimic (20 nM) or scrambled miRNA (20 nM) and either a pcDNA-c-Myc (2 µg) or pcDNA-empty vector (2 µg). (B) Cell proliferation assays with MG-63 cells that were treated as described in (A). (G) Trans-well analyses of MG-63 cells treated as described in (B). The relative ratio of the invasive cells per field is shown. (D) Western blot analyses of c-Myc protein expression in eight patients with miR-135b expression that was down-regulated in the osteosarcoma tissues (C) compared to the corresponding adjacent non-neoplastic tissues (N). The bars represent the mean±SD (*p<0.05, **p<0.01 and ***p<0.001).

RETRACTED

## Discussion

Most cancer deaths are caused by complications that arise from metastasis. The targeting of metastatic disease is therefore a pivotal anti-cancer strategy [17]. Recent studies have revealed a critical role for miRNAs in tumor invasion and metastasis through the regulation of a variety of genes that are necessary for invasion or metastasis [18]–[20]. In this study, we found that miR-135b expression is down-regulated in osteosarcoma cells and tissues in comparison with paired adjacent non-tumor bone tissues. Statistical analyses revealed that the expression level of miR-135b was significantly correlated with metastasis. In addition, we found that the ectopic expression of miR-135b suppressed osteosarcoma cell proliferation, migration, and invasion in the osteosarcoma cell line MG-63. Furthermore, we also identified c-Myc as a novel and direct target of miR-135b. Our findings suggest that miR-135b has a suppressor role in osteosarcoma tumorigenesis and cancer cell invasion.

Previous studies have shown that miR-135b is required for osteogenic cell development and that it is enriched in the placenta where it regulates the growth rate of placental cells [21], [22]. It has also been reported that miR-135b is involved in the progression of several types of cancer [12]. For example, miR-135b has been found to be overexpressed in colon, breast, and lung cancer [12]–[16]. Thus, we measured the level of miR-135b in four osteosarcoma cell lines and 80 osteosarcoma samples. Our results showed that miR-135b was down-regulated in 71 osteosarcoma cases (71/80, 88.8%) and that the expression of miR-135b in osteosarcoma tissues was significantly lower than in adjacent tissues. We also found that the lower expression of miR-135b in osteosarcoma specimens was correlated with metastasis. All of this evidence indicates that miR-135b may contribute to osteosarcoma malignancy.

Cell transfections were performed to further verify the role of miR-135b in the development of osteosarcoma. The ectopic of miR-135b significantly inhibited cell proliferation, migration and invasion, which indicates that the repression of miR-135b may promote tumor progression in osteosarcoma. These results suggest that miR-135b acts as a tumor-suppressor and that down-regulation of miR-135b may contribute to the progression and metastasis of osteosarcoma. However, the underlying mechanisms of miR-135b are still unclear.

RETRACTED

The multi-step process of tumor invasion and metastasis is complex, and miR-135b may play different roles through regulation of different targets. To explore the molecular mechanism by which miR-135b suppressed osteosarcoma cell growth, migration and invasion, we identified c-Myc as a direct target of miR-135b in osteosarcoma cells. To uncover a putative association between miR-135b and c-Myc expression, luciferase reporter and Western blot assays were performed. A sequence that is complementary to miR-135b was identified in the 3′UTR of the c-Myc mRNA sequence, and overexpression of miR-135b led to a significant reduction in c-Myc expression at the protein level. The overexpression of miR-135b also suppressed the c-Myc 3′UTR luciferase reporter activity, and this effect was abolished by mutation of the miR-135b binding site. These results indicate that miR-135b may function as a tumor suppressor in part by repressing c-Myc expression during the development of osteosarcoma.

c-Myc is a key basic helix-loop-helix leucine zipper transcription factor that acts as an important regulator of several cellular processes, including cell migration, growth and proliferation in various cell types [23]–[25]. Moreover, the c-Myc oncogene is overexpressed in many types of human cancers and contributes to cancer cell cycle progression, cell invasion, migration, metastasis, and angiogenesis [26]–[28]. Furthermore, the overexpression of c-Myc is considered to be a potential or independent predictor of poor prognosis for clinical patients in multiple types of cancer [29]. Previous studies have shown that c-Myc mRNA expression is up-regulated in osteosarcomas in comparison with adjacent pair-matched non-tumor tissues. Survival analyses have indicated that high c-Myc expression was associated with lower disease-specific survival rates than in cases that were negative for c-Myc expression [30]–[33]. However, the underlying mechanisms are unclear. Our data showed that the ability of miR-135b to target c-Myc may be one of the mechanisms that regulate c-Myc at the post-transcriptional level.

In conclusion, the current study provided novel evidence that miR-135b is significantly down-regulated in osteosarcoma clinical specimens and appears to function as a tumor suppressor in osteosarcoma through the regulation of c-Myc expression, cell migration, and cell invasion. The identification of miRNA-mediated tumor-suppressor pathways in human osteosarcoma may provide new information on potential therapeutic targets in the treatment of osteosarcoma.

RETRACTED

## Supporting Information

Table S1 **Clinicopathologic charateristics of patients with osteosarcoma.**
(DOC)

Table S2 **Primer sequence.**
(DOC)
